# The Diagnostic Value of Scanning in the Injury of Triceps Crus of Volleyball Players

This article has been retracted.

**DOI:** 10.1155/2022/2203065

**Published:** 2022-05-23

**Authors:** Jinfeng Zhao, Jianxin Liu

**Affiliations:** Pingdingshan University, Henan, Pingdingshan 467000, China

## Abstract

The study goal is to solve the problem of the diagnosis of triceps crus injury of volleyball players, meet the needs of volleyball players and team doctors for the correct diagnosis of triceps crus injury scanning, make up for the deficiency that triceps crus injury scanning diagnosis is easy to make mistakes, and improve the efficiency and ability of triceps crus injury diagnosis scanning. Because the experiment involves the technical action of volleyball jump serve, DELSYSR Trignomobile wireless portable surface electromyography tester (16 leads) made in the United States is selected to test the surface electromyography of the main muscle groups of college male volleyball players in the process of jump serve. The German made simi-3D motion image system is used to conduct three-dimensional synchronous test of athletes' jump serve action. The data analysis software adopts EMG work analysis, EMG analysis software, and simi-3D motion image analysis system for postprocessing data. The original signal is filtered (400 Hz for low pass and 20 Hz for high pass) and rectified. Finally, IEMG, EMG contribution rate, and RMS were calculated. This ensures the accuracy of the experiment.

## 1. Introduction

In recent years, with the development of sports technology and the continuous improvement of training level, volleyball has gradually developed rapidly in the form of height, speed, strength, technology, and team cooperation and the competition among sports teams is becoming more and more fierce. “Every ball must be fought” has become an important goal for the team to carry out tactics and technology. All volleyball powers in the world have made deliberate research on how to improve the attack of their own team and strengthen the defense ability of the other team [1]. Serving skill is one of the basic skills of volleyball. It is the beginning of volleyball match and the beginning of attack of sports team. As an important offensive way in volleyball competition, serving can effectively destroy the stability of the opponent's first pass, interfere with the opponent's offensive ability, reduce the pressure of blocking or defense, and create favorable conditions for the team's attack. Therefore, with the increasingly fierce and competitive volleyball competition, volleyball service technology has gradually evolved to be more and more aggressive [2].

Although the jump serve has the characteristics of fast ball speed, strong attack interferes with the opponent's rhythm and causes the opponent to receive the ball with a high error rate. However, the jumping service technology has very high requirements for athletes' sports technical level, psychological stability, and physical quality. Relevant research shows that when jumping serve, athletes need to have higher take-off height, higher hitting point, and larger horizontal displacement to ensure greater ball speed. Therefore, the action technical structure of jumping serve is more complex and more difficult than that of in situ serve. This requires athletes to have good explosive power, bouncing power, coordination, and ball control ability. It means that athletes are more likely to be injured. Therefore, the experimental analysis of athletes' triceps injury is carried out. We prepare the experimental equipment, complete the site layout and instrument erection, and set up and calibrate the instrument at the same time [3]. The experimental site is shown in Figure 1.

We conduct a preliminary experiment, inform the selected athletes of the experimental purpose, task, and experimental process, as well as the main precautions in the experimental process, and provide basic information such as athletes' height, weight, age, and position on the field. The basic information of the preliminary research object is shown in Table 1.

The preliminary study is for reference only.

## 2. Literature Review

Zhao et al. said that the core is a whole composed of waist, pelvis, and hip joint, which is the middle link of the human body [4], specifically, from the area below the shoulder joint to the area above the hip joint, including the pelvis, and the muscle groups covered include the back, abdomen, and all the muscle groups constituting the pelvis, with a total of 29. In 1996, Qu et al. first put forward the theory of trunk support force, which may be the earliest statement about core force [5]. In 2005, Sun et al. called the power to improve physical stability core power [6]. Since the 1990s, core strength training has been gradually applied to the field of competitive sports training in the United States. Sun et al. classified the muscles on the chest, back, abdomen, lumbosacral, and hip as core muscles [7]. They believe that the core muscle group not only includes rectus abdominis, transverse abdominal muscle, oblique abdominal muscle, back muscle, lower back muscle, and vertical muscle but also the muscles around the hip joint, and gluteus, hip rotator, and posterior femoral muscle group also belongs to the core muscle group of the human body. Zhu et al. put forward the core strength training method of raising and squatting [8] and analyzed the action essentials and precautions of this training method. It is considered that this training method can promote the coordinated strength of athletes' upper and lower limbs, stimulate the continuous contraction of deep muscles, and recruit more deep small muscles to participate in sports, which plays an important role in improving the balance and stability of the body. Xu et al. established the core strength training method based on the core training theory [9]. The scheme is mainly implemented and completed through four stages. The first stage allows athletes to master the methods of core strength training. The second stage allows athletes to practice slowly in a steady state. The third stage allows athletes to carry out static training in an unstable state. The fourth stage allows athletes to continue dynamic practice in an unstable state and let athletes slowly adapt to and master core strength training in a gradual process and feel the fitness value of core strength training. Yu et al. believe that core strength training can improve the transmission efficiency of strength between athletes' upper and lower limbs [10]. Facco et al. believe that the energy consumption of the upper and lower limbs is reduced during exercise, so as to improve the stability of the trunk [11].

With the increasing intensity of volleyball competition, the requirements of athletes' skills and tactics and various abilities related to competitive level are also increasing. At the same time, physical fitness is a prerequisite for all volleyball skills and has attracted more and more attention from researchers and coaches. An excellent volleyball team must keep coordination and progress in intelligence, psychological quality, volleyball field skills, and basic physical fitness [12]. Among the above five components of competitive ability, physical fitness is the basis and prerequisite for all skill performance. Exquisite technology and tactics can play a full role only with the support of good physical fitness. Without the advantage of physical level, there will be no chance to obtain more advanced competitive skills and field tactics. Therefore, physical factor is very important. It is the prerequisite for the formation of volleyball players' technology and the basis for mastering tactics and playing in the field. The ability of jumping and lower limb movement speed is also highly required in volleyball. At the same time, the arm swing action is required to be fast and powerful, which makes the special physical fitness training of volleyball becomes a hot issue that coaches and researchers have always paid attention to. In volleyball, training or competition on the field, athletes often use movements such as left and right forward and backward movement, bouncing, and arm swing. The mode composed of these three has become the main sports mode of volleyball competition. For volleyball players, the special physical fitness of this sport is the ability to realize the above mode. Specific to the competition process, the special physical fitness is manifested in the movement, bouncing, smashing, blocking, and arm swing of athletes. Therefore, in order to improve the special physical fitness level of volleyball players, the core strategy should be to promote the ability of athletes in the three main movements and improve the strength, explosive level, action quality, action speed, and response sensitivity in the core area [13].

In recent years, the concept and training of core strength have been introduced into various sports. The effect of targeted training is very remarkable and has been popularized and applied in the field of sports training. Core strength first appeared in the field of sports rehabilitation, which is used to maintain the stability of the waist, pelvis, and hip. Each sport has its own core strength. Because in all sports, the coordination between muscle and bone is involved, and a specific central muscle group is connected to form a complete sports chain. In the process of sports, the human body needs to change or maintain a specific posture and transfer limb strength, and the core strength plays a key role in this process. In addition, athletes' learning of technical movements also depends on the core strength to a large extent. The lack of core strength will limit the play of tactics and skills in the field and become the bottleneck of athletes' professional level. The long-term practice in sports training has proved that only when the muscle strength reaches a certain threshold, athletes can realize the skilled operations such as flexibility, sensitivity, endurance, and explosive speed. In order to improve their sports skills and break through the bottleneck of comprehensive level, they need to forge enough muscle strength first. A good foundation of core strength can reduce the probability of sports injury, whether the core strength is sufficient and related to the realization and improvement of special skills and the basic protection of athletes [14].

Although there are still great disputes about the specific positioning of the “core,” most experts and scholars define the position of the “core” around the lumbar spine, pelvis, and hip joint. On the basis of summarizing previous studies, this paper believes that the core is the center of the human body, which refers to the area below the shoulder joint and above the hip joint. It includes all the muscles of the back and abdomen, the deep muscles attached to the spine and around the hip joint, and all the muscle groups constituting the pelvis.

## 3. Method

### 3.1. Sports Injury

There is no unified standard for the definition of the concept of “sports injury.” Scholars believe that the definition of injury depends on the time for athletes to receive sports guidance or rehabilitation, while some scholars believe that there are only two views on the effect of sports training on injury [15]. Gait is the behavior characteristic of human walking, which is affected by many factors. The control of walking is very complex, involving the coordinated movement of all joints and muscles of the whole body. The imbalance of any link may affect walking and gait, and the abnormality may also be compensated or covered up. After sports injury, the most obvious symptom is pain, which has a significant impact on gait. Pain is easy to lead to the shortening of gait support phase time and the prolongation of swing phase on the injured side. Hahn et al. concluded that the support phase time of patients with unilateral knee injury is shorter than that of patients without injury, so as to reduce the load of knee joint on the injured side, while the support phase time of patients with bilateral knee injury is prolonged, so as to increase the time of double support phase and reduce the load on one side of knee joint alone. Studies of patients with increased proprioceptive pain of the knee joint (and of patients with increased proprioceptive pain of the knee joint) seem to point out that the purpose of the study is to reduce the abnormal gait [16]. Many people have studied the time distribution of plantar pressure and ground vertical reaction force in patients with knee osteoarthritis (KOA). It is pointed out that due to pain, the time of single foot bearing period on the injured side of KOA patients is shortened, so as to reduce the time for the injured side to support weight alone. In addition, the pain will also make the heel dare not touch the ground, and the leg is weak when the foot is off the ground. Some studies have pointed out that the foot pressure center of gravity of athletes with repeated foot and ankle injury tends to shift to the front area of the foot, the time of front foot support is prolonged, and the time of rear foot support is reduced, which may be the protective mechanism adopted to reduce the load of foot and ankle joint on the injured side [17, 18].

Time domain characteristics regard muscle tone signal as a function of time, which can reflect the statistical characteristics of muscle tone signal in time domain. And because the calculation of time-domain characteristics does not need any conversion, it can be calculated directly from the original muscle tone signal sequence. Therefore, the calculation method is simple and the calculation speed is fast, which has been widely used in the field of signal analysis.

#### 3.1.1. IMMG

IMMG is obtained by integrating the time series of muscle tone signal, and its expression is shown in

(1) $$\begin{array}{c} \text{IMMG}=\frac{\sum_{i=1}^{N}\left|xi\right|}{N}. \end{array}$$

#### 3.1.2. MAV

MAV is the absolute mean value of muscle tone signal amplitude, and its calculation formula is shown in

(2) $$\begin{array}{c} \text{MAV}=\frac{1}{n}\overset{N}{\underset{i=1}{\sum }}\left|xi\right|. \end{array}$$

#### 3.1.3. MAVI

MAVI is an extension of MAV. The introduction of weighted window function can improve the robustness of features. Its expression is shown in

(3) $$\begin{array}{c} \text{MAVI}=\frac{1}{n}\overset{N}{\underset{i=1}{\sum }}wi\left|xi\right|. \end{array}$$

#### 3.1.4. SSI

SSI represents the energy of muscle tone signal, and its calculation formula is shown in

(4) $$\begin{array}{c} \text{SSI}=\overset{N}{\underset{i=1}{\sum }}{xi}^{2}. \end{array}$$

#### 3.1.5. VAR

VAR represents the degree to which the signal deviates from the average value, and its expression is shown in

(5) $$\begin{array}{c} \text{VAR}=\frac{1}{N-1}\overset{N}{\underset{i=1}{\sum }}{\left(xi-\bar{x}\right)}^{2}. \end{array}$$

#### 3.1.6. TM3, TM4, and TM5

These three feature lengths are used for classification research, which can reduce the intra class interval. The calculation formula is shown in

(6) $$\begin{array}{c} \text{TM}3=\left|\frac{1}{N}\overset{N}{\underset{i=1}{\sum }}{xi}^{3}\right|,\\ \text{TM}4=\left|\frac{1}{N}\overset{N}{\underset{i=1}{\sum }}{xi}^{4}\right|,\\ \text{TM}5=\left|\frac{1}{N}\overset{N}{\underset{i=1}{\sum }}{xi}^{5}\right|. \end{array}$$

#### 3.1.7. RMS

RMS represents the amplitude value at the maximum probability density of the signal, and its calculation formula is shown in

(7) $$\begin{array}{c} \text{RMS}=\sqrt{\frac{1}{N}\overset{N}{\underset{i=1}{\sum }}{xi}^{2}}. \end{array}$$

#### 3.1.8. LRMS

LRMS is similar to RMS and further enlarges the spacing between features. Its expression is shown in

(8) $$\begin{array}{c} \text{LRMS}=\log\left(\text{RMS}\right). \end{array}$$

Frequency domain characteristics are helpful to analyze the signal in frequency domain and understand the characteristic change trend of the signal in power spectrum. They are mainly used in the supplementary analysis of muscle fatigue and motor units. For the frequency domain analysis of muscle tone signal, firstly, the power spectrum of the signal needs to be obtained by Fourier transform, and the power spectral density is calculated. Then, the frequency domain characteristics of the signal are obtained by statistical method.

### 3.2. Relationship between Sports Injury and Stride Length

Stride length is another important parameter in gait characteristics. Stride length was significantly correlated with height. Generally speaking, the height is higher and the stride is longer. The stride length of female special students was significantly larger than that of ordinary female college students, and there was no significant difference between the two after standardization by dividing the stride length by height (female special students 0.76 ± 0.07, ordinary female college students 0.75 ± 0.05, *P* > 0.05). This shows that the stride difference between female special students and ordinary female college students may be related to height. Studies have shown that college students who often participate in physical exercise have fully developed their lower limb muscle strength and stability, so that the stride step of college students who participate in physical exercise for a long time is significantly larger than that of college students who do not participate in physical exercise. The height of male special students is significantly higher than that of ordinary male college students. At the same time, they also participate in sports training for a long time, and their physical quality and sports ability have been improved to varying degrees. However, there is no significant difference in stride between male special students and ordinary male college students. After standardization by dividing stride by height, there is still no significant difference between the two (male special students 0.73 ± 0.08, ordinary male college students 0.77 ± 0.02, *P* > 0.05). This shows that the stride characteristics of male students may be related to volleyball [19].

Many scholars pointed out in their research that the sagittal range of motion of the hip joint is the main factor affecting stride. The range of motion of the hip joint in sagittal plane is positively correlated with walking speed, and the range of motion of the hip joint and knee joint in sagittal plane increases with the increase of walking speed. Step length, stride length, and step frequency also increase with the increase of step speed. The walking speed of male special students is significantly lower than that of ordinary male college students. The walking speed is small, and the motion range of hip joint in sagittal plane is reduced, which may lead to the shortening of stride. In this study, the height of male special students is significantly higher than that of ordinary male college students, and there is no significant difference in stride between male special students and ordinary male college students, which may be related to the slow pace and insufficient hip flexion of male special students.

Hip joint is an important joint connecting the trunk and lower limbs, with complex structure and more weight-bearing. Hip joint not only supports the stability of human body upright but also coordinates the center of gravity of the body in the process of movement. It is one of the indispensable joints to maintain human body stability and complete body movements. Good hip flexion ability can improve sports performance and daily activity ability. The improvement of hip flexion flexibility can improve athletes' speed, strength, and explosive power to varying degrees. However, if hip flexion is limited, it may cause pain in other parts of the body, such as the back or knee, because many movements of the body need the cooperation of multiple joints, such as bending, which needs the cooperation of the lumbar spine, thoracic spine and hip joint. If the flexion of hip joint is limited, it will force the lumbar spine and thoracic spine to increase their range of motion to compensate for the reduced flexion range of the hip joint, so as to increase the risk of sports injury in other parts [20].

The stride characteristics of male special students may be related to their insufficient hip flexion. Therefore, after strength training of hip extensor group in daily training, pay attention to fully stretch and relax the hip extensor group to avoid excessive tension of extensor group. At the same time, we also need to strengthen the strength training of hip flexor group, improve the flexion ability of hip joint, improve sports performance, reduce the risk of hip joint injury, and avoid the injury of waist or chest caused by compensatory hip joint flexion limitation.

## 4. Results and Analysis

Before the test, the questionnaire was distributed to the subjects on site, and the subjects filled it out on site. After filling it out, the researchers asked about the questionnaire and the actual situation of the subjects and recorded the inquiry results on the questionnaire [21]. The statistics of questionnaire distribution and recovery are shown in Table 2.

The gait data of the subjects are exported in Excel form from the gait view software, and the recovered sports injury investigation data are systematically classified and sorted. The data and data obtained from the investigation and test are processed and statistically analyzed with spss160, and the statistical results are expressed in the form of mean ± standard deviation (M ± SD) and histogram.

*T*-test was mainly used for the mean difference of gait parameters, and the significance level of *P* value was 0.05.

A total of 64 volleyball special students (experimental group) participated in the test, including 42 male special students and 22 female special students; a total of 40 ordinary college students (control group) participated in the test, including 22 boys and 18 girls, see Table 3 for the basic information of the subjects in the experimental group and the control group.

It can be seen from Table 3 that compared with female students, the male students involved in the test have the same age (*P* > 0.05), there is no significant difference in the years of Volleyball (*P* > 0.05), and there is a very significant difference in height and weight (*P* < 0.01). Compared with female college students, ordinary male college students are also the same age (*P* > 0.05), and there are very significant differences in height and weight (*P* < 0.01).

Compared with ordinary male college students, male special students are of the same age. The height and weight of male special students are significantly higher than those of ordinary male college students (*P* < 0.01). Compared with ordinary female college students, female special students are also the same age, and their height and weight are significantly higher than ordinary female college students (*P* < 0.01).

Before the gait test, the sports injuries of 64 volleyball special students were investigated, and the sports injuries of volleyball special students were counted. Among the 64 volleyball students, 53 had sports injuries, and the injury rate was as high as 82.81%. 37 male students had a history of sports injury, and the incidence of injury was 88.10%. There were 16 female students with a history of sports injury, and the incidence of injury was 72.73%. There was no significant difference in the incidence of sports injury between male and female students (*P* > 0.05), see Table 4. The triceps injury of lower leg is shown in Figure 2.

The results of this experiment show that there is no significant correlation between the incidence of waist injury and height and weight of volleyball students (*P* > 0.05), and there is a significant correlation with the number of years of exercise (*P* < 0.05). Therefore, it can be inferred that long-term high-intensity exercise training is one of the causes of waist injury [22].

Volleyball players often need to bend over, fish jump, roll over, and fall to the ground to save the ball. They have high speed, high intensity, and high requirements for body control. Therefore, the pressure on the waist is large, which is easy to cause pain or acute injury in the waist [23]. In addition, the requirements of serving and spiking on the waist and back muscles are quite high, which requires good muscle strength and explosive power in the waist and abdomen, and the intensity and amplitude of lumbar activity are overloaded, which is very easy to produce lumbar injury. When completing other basic technical movements of volleyball, the lumbar and abdominal muscles should also participate in work. In long-term heavy-load training and competition, the muscles and ligaments around the waist are prone to excessive fatigue. If they are not reasonably relaxed and rested, it is easy to cause chronic lumbar strain or aggravate the strain. The longer the years of sports training, the higher the risk of chronic lumbar strain [24].

In addition, insufficient preparation activities, incorrect take-off and landing movements, unstable landing, loss of center of gravity, insufficient strength of supporting legs when landing, no buffer on landing, increased impact on the waist, incorrect action during barbell strength training, unbalanced development of abdominal and back muscle strength, etc. are also easy to induce lumbar injury. Once the waist injury occurs, it is not easy to completely cure it. If the waist injury is not cured, training or competition will be arranged, and the injured part will not be well treated and recovered. In the long run, chronic strain will form, and the impact on the body will be more serious, forming a vicious circle [25].

Intervertebral disc is a fibrocartilage disc located between adjacent vertebral bodies, which has great elasticity and toughness. Due to the existence of intervertebral disc, the spine can perform forward flexion, backward extension, and lateral flexion [26]. The human lumbar intervertebral disc is the thickest, and the articular surface of the lumbar facet is almost sagittal, so the flexion and extension activities of the waist are flexible, but the rotation movement of the waist is limited, and the axial rotation range of the waist is small, only 5°. However, the overall range of axial rotation of the waist is large, which is due to the cooperative rotation of the thoracic spine and hip joint. In volleyball, the basic technique commonly used by athletes is cushion, which is the main technical action in receiving, defending, and dealing with all kinds of difficult balls. In the cushion action, the athlete needs to straighten and clamp his arms and close his abdomen with his chest. Such technical action basically locks the chest, thus limiting the axial rotation range of the chest. At the same time, when volleyball players do various technical movements, they are often in the hip flexion position, the hip joint is relatively fixed, and the axial rotation range of the hip joint is also relatively reduced. However, in volleyball, there is a high demand for the axial rotation range of the body. If the axial rotation range of the chest and hip joint is reduced, the pressure on the lumbar muscles and joints will increase, thus increasing the risk of lumbar injury. Therefore, it is necessary to increase the stretching activity of chest muscles in daily training to fully relax the chest in a state of tension for a long time [27].

In this experiment, the most damaged part of female students is the waist, which may be related to the physiological characteristics of women. The periodic changes of estrogen and progesterone levels in women have a certain impact on the joints and ligaments of women; when the estrogen level of women's body is high, the joint ligaments are relatively loose. If girls' waist is trained with high intensity during this period, it is easy to cause lumbar injury.

The experimental results show that the left side is significantly larger than the right side in the unilateral lumbar injury, suggesting that the pressure on the left waist of volleyball students may be greater than that on the right side, which should be paid attention to accordingly. Volleyball special students keep bending posture for a long time, the waist burden is too heavy, and the muscle tension increases, which destroys the coordination of lumbar muscles, reduces the elasticity and toughness of lumbar muscles, and will cause lumbar muscle strain for a long time. In volleyball, the technical actions such as serving and spiking often require waist rotation. Repeated and single special movement training makes the lumbar muscles frequently squeezed or pulled, and the local training intensity is too large, which is easy to lead to lumbar injury on one or both sides [28].

## 5. Conclusion

It is proved that it is feasible to apply the calculation of time-domain characteristics to the diagnosis of triceps crus injury of volleyball players. It can effectively solve the problem of cumbersome diagnosis of triceps crus injury of volleyball players, meet the needs of rapid diagnosis of sports injury of professional volleyball players, make up for the lack of slow diagnosis of sports injury before, and improve the efficiency of timely detection of volleyball players after injury. In this experiment, the right hand is the favorable hand of most volleyball students. When serving and spiking, the waist needs to exert force to drive the arm to turn to the right, and the left waist is prone to injury due to long-term extrusion, which may be one of the reasons why the left waist injury of volleyball students is significantly greater than that of the right.

## Figures and Tables

**Figure 1:** Experimental site.

**Figure 2:** Distribution of triceps injury of the lower leg.

**Table 1:** Basic information of preliminary research objects.

Gender	Quantity	Age (years)	Height (cm)	Weight (kg)	Training years
Experience group	10	21.6 ± 2.2	187.7 ± 4.5	78.5 ± 4.6	8.4 ± 3.1

**Table 2:** Statistical table of injury questionnaire.

Survey object	Distribution (copy)	Recycling (copies)	Valid questionnaire	Recovery rate (%)	Effective rate (%)
Volleyball students	64	64	64	100	100

**Table 3:** Basic information of subjects (m ± SD).

Grouping	Gender	Number of people	Age (y)	Height (cm)	Weight (kg)	Years of professional sports (y)
Experimental group (*N* = 64)	Male	42	20.02 ± 1.14	184.00 ± 6.09^∗∗^	74.57 ± 8.93^∗∗^	6.31 ± 1.89
	Female	22	19.64 ± 1.33	172.55 ± 7.31^##^	61.91 ± 9.12^##^	6.14 ± 1.96
Control group(*N* = 64)	Male	22	20.12 ± 0.93	170.00 ± 4.82^##^	61.88 ± 7.O9^##^	—
	Female	18	19.77 ± 0.73	160.69 ± 5.14^∗∗^	49.31 ± 6.36^∗∗^	—

**Table 4:** Injury rate of special students of different genders in the injury group.

Gender	Number of injured	Number of people without injury	Damage rate (%)
Male	37	5	88.10
Female	16	6	72.73
Total	53	11	82.81

## Data Availability

The data used to support the findings of this study are available from the corresponding author upon request.
